# GNA13 promotes tumor growth and angiogenesis by upregulating CXC chemokines via the NF‐κB signaling pathway in colorectal cancer cells

**DOI:** 10.1002/cam4.1783

**Published:** 2018-09-28

**Authors:** Zhongqiang Zhang, Xiao Tan, Jing Luo, Beibei Cui, Sanlin Lei, Zhongzhou Si, Liangfang Shen, Hongliang Yao

**Affiliations:** ^1^ Department of General Surgery The Second Xiangya Hospital Central South University Changsha Hunan China; ^2^ Department of Oncology Xiangya Hospital Central South University Changsha Hunan China

**Keywords:** CRC, CXCL chemokines, GNA13, NF‐κB

## Abstract

GNA13 has been found overexpressed in various types of cancer, which is related to tumor metastasis and progression. However, the biological functions of GNA13 in colorectal cancer (CRC) progression remain unclear. This study aimed to explore the role of GNA13 in CRC and investigate the mechanism of how GNA13 promotes tumor growth. Interestingly, our findings showed that GNA13 is commonly upregulated in CRC, where these events are associated with a worse histologic grade and poor survival. Increased expression levels of GNA13 promoted cell growth, migration, invasion, and epithelial‐mesenchymal transition, whereas GNA13 silencing abrogated these malignant phenotypes. In addition, overexpressing GNA13 in cancer cells increased the levels of the chemokines CXCL1, CXCL2, and CXCL4, which contributed to CRC proliferation and colony formation. Moreover, our mechanistic investigations suggest that the NF‐κB/p65 signaling pathway was activated by the increase in GNA13 levels. Inhibiting the NF‐κB/p65 pathway with an inhibitor decreased GNA13‐induced migration, invasion and CXCL chemokine level increases, indicating the critical role of NF‐κB/p65 signaling in mediating the effects of GNA13 in CRC. Together, these results demonstrate a key role of GNA13 overexpression in CRC that contributes to malignant behavior in cancer cells, at least in part through stimulating angiogenesis and increasing the levels of the NF‐κB‐dependent chemokines CXCL1, CXCL2, and CXCL4.

## 1 INTRODUCTION

Colorectal cancer (CRC) is one of the most frequently diagnosed types of cancer, and it is the third most common contributor to cancer‐related deaths in the United States.^1^ Various biomarkers have been shown to be involved in the progression of CRC.^2^, ^3^ The identification and verification of prognostic factors can improve the treatment as a complement to clinical histopathology.

G protein‐coupled receptors (GPCRs) are the largest and most diverse family of cell surface receptors in eukaryotes.^4^ GPCRs interact with G proteins, which are composed of three different subunits: the Gα subunit, the Gβ subunit, and the Gγ subunit.^5^ The α subunits of G proteins are divided into four subfamilies: Gs, Gi, Gq, and G12.^6^ Among them, the G12 protein comprises Gα12 (GNA12) and Gα13 (GNA13) and plays a critical role in promoting cancer cell growth and oncogenic transformation.^7^, ^8^ Previous studies have implicated that GNA12 proteins crucially regulate dorsal ruffle turnover, which is involved in an incredible array of functions, including tumor cell invasion, micropinocytosis, metastasis, and others.^9^, ^10^ However, there are more studies that have focused on the role of GNA12 in cancer biology, but few have studied the specific role of GNA13.^11^ Recently, the upregulation of GNA13 was reported in several malignant neoplasms, such as aggressive prostate, breast, and pancreatic cancers.^12^, ^13^ Moreover, highly increased expression levels of GNA13 could cause invasive and migratory effects in breast cancer cells.^12^, ^14^ Previous studies have indicated that increased expression levels of GNA13 play a critical role in the tumorigenicity and proliferation of gastric cancer cells.^15^ However, the effects and role of GNA13 expression levels in colon cancer cells remain unknown.

In this study, we aimed to determine the role of GNA13 in CRC. We investigated the effects of the overexpression of GNA13 on the expression of multiple chemokines in CRC. We further explored how NF‐κB inhibition affected the expression of chemokines induced by GNA13.

## 2 MATERIALS AND METHODS

### 2.1 Cell culture and reagents

The human CRC cell lines HCT116 and HT29 were procured from the American Type Culture Collection (ATCC, Manassas, VA, USA) and were cultured in RPMI‐1640 medium supplemented with 100 μg/mL streptomycin, 100 units/mL penicillin, and 10% heat‐inactivated newborn calf serum (Invitrogen, Carlsbad, CA, USA). Cell lines were tested for mycoplasma every 6 months using a MycoAlert Detection Kit (Lonza, Walkersville, MD, USA).

### 2.2 IHC (Immunohistochemistry)

Human CRC tissue microarrays (paraffin‐embedded), including follow‐up survival information, were provided by SuperBioChips. The arrays underwent incubation with an anti‐GNA13 antibody (1:200) in a solution of 0.1% Triton X‐100 and 5% bovine serum albumin/PBS (Sigma, St. Louis, MO, USA) for 16 hours at 4°C. Then, the fixed cells were incubated in 0.1 mol/L Tris‐HCl, pH 7.5, containing 0.05 mol/L acetic acid (chondroitinase reaction buffer) and 0.5 units/mL protease‐free chondroitinase ABC (Sigma) for 2 hours at 37°C. The immunostaining was observed using 3,3‐diaminobenzidine and hematoxylin (Sigma) counterstain and an UltraVision Quanto Detection System (Thermo Fisher Scientific Inc, Pittsburgh, PA, USA). The distribution and positive intensity of GNA13 were analyzed by two individuals according to a double‐blind experimental design. The staining scores were given according to the percentage of positive tumor cells (0, 0%; 1, <25%; 2, 25%‐50%; 3, 51%‐75%; and 4, >75%) and staining intensity (0, none; 1, weakly stained; 2, moderately stained; and 3, strongly stained).

### 2.3 Quantitative real‐time PCR

Total RNA was separated using TRIzol reagent (Invitrogen). One microgram of total RNA was used for reverse transcription reactions using a PrimeScript™ RT Reagent Kit (TaKaRa, Dalian, Liaoning, China). Real‐time PCR was performed on the cDNA. The specificity of amplification by the primers was confirmed by sequencing the PCR products.

### 2.4 Transfection

For the overexpression experiments, GNA13 cDNA was subcloned into pcDNA3.1 vector. Cells were transfected with plasmids using Lipofectamine 2000 (Invitrogen). The pcDNA3.1 plasmid was used as a control. The transfected cells were selected with 5 μg/mL G418 for 2 weeks. For the shRNA knockdown experiments, two pLKO/GNA13‐shRNA plasmids were obtained from Santa Cruz Biotechnology (Dallas, TX, USA). The short hairpin RNA (shRNA) plasmids were transfected and selected using 3 μg/mL puromycin for 2 weeks.

### 2.5 Western blotting

Western blotting was performed as described previously^16^ with antibodies against LOX, MMP2, MMP9 (Cell Signaling Technology, Beverly, MA, USA), ZO‐1, vimentin, VEGF, β‐actin (Abcam, Shanghai, China), β‐catenin, cyclin D1, c‐myc, MMP7, and p‐GSK3β Ser9 (Santa Cruz Biotechnology, Dallas, TX, USA).

### 2.6 Cell proliferation and colony formation

Indicated cells (4 × 10^4^) were seeded into 96‐well plates with culture medium. An analysis of viable cells at 72 hours was carried out using an MTS assay. For the anchorage‐dependent colony formation assay, 500 cells were seeded in 6‐well plates and incubated for 2 weeks. The colonies were fixed in methanol and stained with 0.1% crystal violet (Sigma) before counting.

### 2.7 Cell migration and invasion assay

Transwell inserts with porous filters without coats (the pore size was 8 μm) for 24‐well plates were used for evaluating cell migration, and Matrigel (BD Biosciences, Franklin Lakes, NJ, USA) porous filters with coats were used for examining cell invasion. First, 2 × 10^4^ cells in serum‐free DMEM (0.2 mL) were seeded onto the inserts; then, 0.6 mL of DMEM with 10% FBS was added to the lower portion of the well.

### 2.8 Enzyme‐linked immunosorbent assay (ELISA)

Using ELISA kits (RayBiotech, Norcross, GA, USA), we quantified CXCL4 and CXCL1 protein levels in the supernatants of HCT116 and HT29 cells that stably expressed control shRNA or shRNA against GNA13 and were cultured in control media for a day.

### 2.9 Endothelial cell tube formation assay

Primary human umbilical vein endothelial cells (HUVECs, Life Technologies, Carlsbad, CA, USA) were cultured in 200PRF medium. Trypsinized HUVECs were then suspended in conditioned media, seeded on Matrigel (Corning, Corning, NY, USA) with reduced concentrations of growth factors for 24 hours, and labeled with CMFDA (5‐chloromethylfluorescein diacetate; Life Technologies). The cells were photographed four times at random. The lengths of the tubes were measured at 40X magnification with Zeiss AxioVision software and expressed as mm/mm^2^.

### 2.10 Xenograft models

The experiments involving animal subjects in this study were conducted in accordance with the internationally accepted principles for laboratory animal use and care. The study was approved by the Committee on the Ethics of Animal Experiments of Xiangya Hospital, Central South University. For tumor growth analysis, 5 × 10^6^ HCT116 mock transfectants were injected subcutaneously into the left flanks of nude mice, and an equal number of GNA13 transfectants were injected into the right flanks (n = 6). The tumor volumes were observed for 21 days, and the excised tumor tissues were weighed and analyzed by immunohistochemistry. The surgically removed tissues were paraffin‐embedded for subsequent experiments.

### 2.11 Statistical analysis

Statistical analyses were carried out using GraphPad Prism IV software. *P* values were calculated by Student's *t* test and were considered significant if *P* < 0.05. The means ± 1 standard deviation (SD) is displayed in the figures.

## 3 RESULTS

### 3.1 GNA13 expression is frequently upregulated in CRC and correlates with poor survival

First, we compared the mRNA levels of GNA13 in CRC tissues and paired normal tissues by quantitative real‐time PCR (qRT‐PCR). Notably, CRC tissues had significantly higher expression levels of GNA13 than the paired normal tissues (Figure 1A). Next, we randomly chose 5 paired tissue samples to assess GNA13 protein levels by Western blotting. We found the protein levels of GNA13 were increased in the CRC samples (Figure 1B). These results were confirmed by immunohistochemistry. GNA13 was highly expressed in almost every cancer tissue sample compared to the nontumor tissue samples (Figure 1C). Our results also showed that CRC patients with disease recurrence had higher levels of GNA13 mRNA expression than patients without recurrence (Figure 1D). In addition, for patients with and without metastasis, the GNA13 mRNA level was considerably higher in CRC tissues of patients with metastasis (Figure 1E). To determine whether GNA13 was correlated with the clinicopathological characteristics, GNA13 expression was categorized as high expression (staining index >6) or low expression (staining index ≤6). Interestingly, the results revealed that GNA13 was highly expressed in 54.2% (39/74) of CRC tumors, whereas only 28.5% (2/7) of nontumor tissues expressed high levels of GNA13. According to the Kaplan‐Meier survival analysis, the survival rate of CRC patients who had high GNA13 expression was dramatically lower than the survival rate of those who had low GNA13 expression (Figure 1F). These data indicate that GNA13 is frequently upregulated in colon cancer and that its expression is associated with a high histology grade and poor prognosis.

**Figure 1:** GNA13 is overexpressed in CRC and its overexpression in associated with poor prognosis. A, The mRNA level of GNA13 in CRC tissues (Tumor) and paired normal tissues (Normal) was analyzed by real‐time RT‐PCR. B, GNA13 protein level in CRC tissues and paired normal tissues was assessed by Western blotting. C, Immunohistochemistry of GNA13 in nontumor and primary CRC tissue arrays containing 74 cases. D, Relative mRNA expression of Six1 in HCC samples from patients with disease recurrence (n = 22) or without disease recurrence (n = 23). E, Relative mRNA expression of Six1 in HCC samples from patients with metastasis (n = 19) or without metastasis (n = 22). F, Kaplan‐Meier analysis of overall survival for patients with CRC. The analyses were conducted based on the immunohistochemistry of GNA13 and the survival information provided by the supplier

### 3.2 GNA13 regulates malignant phenotypes and epithelial‐mesenchymal transition in CRC cells

To explore the effects of GNA13 on malignant phenotypes in CRC cells, we analyzed colony formation, cell growth, invasion, and migration. As shown in Figures 2A and 3B, knocking down GNA13 significantly reduced cell proliferation in HCT116 cells, whereas overexpressing GNA13 led to enhanced proliferation. In addition, overexpression of GNA13 enhanced proliferation in LoVo cells (Figure S1A). However, downregulation of GNA13 suppression of cell proliferation in Caco2 cells (Figure S1B). Consistently, overexpressing GNA13 increased the number of anchorage‐dependent colonies, whereas knocking down GNA13 slightly decreased the number of colonies (Figures 2B and 3A). Interestingly, invasion and migration were dramatically promoted by the overexpression of GNA13, and invasion and migration were decreased by GNA13 knockdown. (Figure 2C,D). As we know, cell invasion and morphological changes are tightly associated with epithelial‐mesenchymal transition (EMT). We then examined the expression of epithelial markers, such as E‐cadherin and ZO‐1, and the mesenchymal marker vimentin by Western blotting. These results strongly suggest that overexpressing GNA13 suppressed ZO‐1 and E‐cadherin expression and increased vimentin expression in HCT116 cells. In contrast, knocking down GNA13 enhanced E‐cadherin and ZO‐1 expression but decreased vimentin expression in the cells (Figure 2E). Together, these data indicate that GNA13 can not only modulate CRC cell growth but also regulate colony formation, migration, invasion, and EMT in vitro.

**Figure 2:** Effects of GNA13 on malignant phenotypes in CRC cells (A) Cell viability of HCT116 cells was analyzed by MTS assays at different time points. B, Effects of GNA13 on anchorage‐dependent colony formation. (C) GNA13 regulated Transwell cell invasion and (D) Matrigel invasion. E, Expression of epithelial markers, E‐cadherin and ZO‐1, and mesenchymal markers, vimentin, was analyzed by Western blotting. *, *P *<* *0.05

**Figure 3:** Reduced endothelial cell tube formation upon GNA13 suppression and CXCR2 inhibition. A, After 48 h of the transfection of HCT116 and HT29 cells with GNA13 or vector, mRNA expression of CXCL1, CXCL2, and CXCL4 was quantified by qRT‐PCR (right); GNA13 protein expression was quantified by Western blotting (left). B, Expression of CXCL1, CXCL2, and CXCL4 mRNA in HT29‐GNA13 shRNA, HT29‐control shRNA, HCT116‐GNA13 shRNA, and HCT116‐control shRNA cells was analyzed by qRT‐PCR. C, Amount of CXCL1 and CXCL4 proteins in cell culture supernatants was determined by ELISA after 24‐hour culture of HCT116 and HT29 cells that stably expressed control shRNA or shRNA against GNA13 in a serum‐free media. D, Left: HUVEC tube formation after HUVECs were incubated on Matrigel for 8 h in the conditioned media from 24‐hour culture of HCT116 and HT29 cells that stably expressed control shRNA or shRNA against GNA13 in a serum‐free media. E, Left: the inhibition of HUVEC tube formation by CXCR2 antagonists. The HUVECs were incubated on Matrigel for 8 h in a mixture of AZD5069 or DMSO with the conditioned media from 24‐hour culture of HCT116 and HT29 cells. *, *P *<* *0.05

### 3.3 GNA13 upregulates CXCL1, CXCL2, and CXCL4 to promote tumor angiogenesis

Pro‐angiogenic factors, such as vascular endothelial growth factor, are actively released by tumor cells to promote endothelial cell survival, migration, and proliferation to form new vessels. We further investigated the effects of its overexpression on the expression of CXCL1, CXCL2, and CXCL4. Overexpressing GNA13 in HCT116 and HT29 cells after transfection with the GNA13 plasmid considerably increased CXCL1, CXCL2, and CXCL4 mRNA levels compared to those in the mock‐transfected cells (Figure 3A). Conversely, the mRNA levels were significantly reduced in HCT116 and HT29 cells expressing shRNA against GNA13 compared with those in the cells expressing control shRNA (Figure 3B). Moreover, we observed significantly lower protein levels of CXCL4 and CXCL1/2 in HCT116 and HT29 cells with stable GNA13 knockdown than those in the corresponding control cells expressing shRNA (Figure 3C). Collectively, our results suggest that the overexpression of GNA13 in CRC cells increases CXCL1, CXCL2, and CXCL4 levels.

In the tube formation assay that utilized HUVECs and Matrigel, tube formation was induced in the conditioned media of CRC cells expressing shRNA (control) but not in that of cells with stable GNA13 suppression (Figure 3D). We further clarified the effects of CXCL1, CXCL2, and CXCL4 on HUVEC tube formation by blocking their common signaling receptor CXCR2 with the antagonist AZD5069. HUVEC tube formation was abolished by CXCR2 blockade in the conditioned media of HCT116 and HT29 cells (Figure 3E), indicating that the levels of CXCL1, CXCL2, and CXCL4 induced by GNA13 in CRC cells might promote tumor angiogenesis by binding with CXCR2 receptors on endothelial cells.

### 3.4 GNA13 induces CXCL1, CXCL2, and CXCL4 through the IKKβ/NF‐κB pathway

The autocrine effects of CXCL1 and CXCL4 are important for the survival and proliferation of other types of cancer cells. Transfection of shCXCL1/2 and shCXCL4 into HCT116 and HT29 cells successfully suppressed CXCL1, CXCL2, and CXCL4 expression and resulted in suppressed clonogenic growth and cell proliferation (Figure 4A‐C), suggesting that these three chemokines could promote survival and proliferation in an autocrine manner in CRC cells that overexpress GNA13.

**Figure 4:** GNA13 induces CXCL2, CXCL1, and CXCL4 expression through the IKKβ‐NF‐κB pathway. A, HCT116 and HT29 cervical cancer cells were transfected with CXCL1/2, CXCL4, or control shRNA; after 48 h of transfection, expression of CXCL1, CXCL2, and CXCL4 was quantified by qRT‐PCR. B, In the EdU incorporation assay, 2 d after transfection, reduced expression of CXCL1, CXCL2, or CXCL4 due to shRNAs inhibited HT29 and HCT116 cell proliferation compared with that in the cells transfected with control shRNA. C, Suppression of CXCL1, CXCL2, or CXCL4 by shRNAs inhibits the clonogenic growth of HCT116 and HT29 cells. D, Expression of CXCL1, CXCL2, and CXCL4 mRNA in HCT116 and HT29 cells treated with 2 μm IKKβ inhibitor Bay 65‐1942 or the control was analyzed by qRT‐PCR. E, IKKβ and NF‐κB p65 protein expression was quantified by Western blotting. F, HT29 and HCT116 cells were transfected with shRNA against IKKβ, NF‐κB p65, or the control, after 48 h of transfection, and then expression of CXCL1, CXCL2, and CXCL4 mRNA was quantified by qRT‐PCR. *, *P *<* *0.05

Previous studies suggest that the expression of CXCL1, CXCL2, and CXCL4 is regulated by IKKβ in ovarian cancer cells.^17^ After incubation with inhibitors against IKKβ or p65 for 6 hours, the mRNA expression levels of CXCL1, CXCL2, and CXCL4 in HCT116 and HT29 cells were significantly reduced (Figure 4D). HCT116 and HT29 cells with suppressed IKKβ or p65 expression (mediated by shRNAs that targeted both NF‐κB p65 and the IKKβ subunit) exhibited decreased CXCL1, CXCL2, and CXCL4 mRNA expression levels compared with HCT116 and HT29 cells transfected with control shRNA (Figure 4E,F). Following GNA13 transfection, nuclear fractionation was used to detect p65 translocation. IKKβ inhibitor blocked p65 nuclear translocation (Figure S2). These results demonstrate that CXCL1, CXCL2, and CXCL4 expression induced by GNA13 might be closely correlated with the IKKβ‐NF‐κB signaling pathway.

### 3.5 GNA13 increases tumor growth in vivo

To evaluate the effects of GNA13 on tumor growth, we established a subcutaneous xenograft tumor model in BALB/c nude mice. On the 21st day after inoculation, the tumor volume in the sh‐GNA13 group was decreased compared with that in the shRNA‐con group; the tumor volume in the GNA13 group was larger than that in the vector group, and no tumor volume differences were found between the shRNA‐con and vector groups (Figure 5A). Compared to the shRNA‐con group, the tumor weight in the sh‐GNA13 group was lower, and the tumor weight in the GNA13 group was higher. There were no differences in the tumor weights between the siRNA‐con and vector groups (Figure 5B). The expression of GNA‐13 in tumor was determined by Western blotting (Figure 5C). Immunohistochemistry analyses showed that GNA13 knockdown dramatically decreased cancer cell proliferation, as revealed by Ki67 staining, while GNA13 promoted cancer cell proliferation (Figure 5D).

**Figure 5:** GNA13 enhanced tumor growth in vivo (A) Tumor volume in each group. B, Tumor weight in each group. C, The expression of GNA13 in each group was detected by Western blotting. D, Expression of Ki‐67 (cell proliferation marker) in xenograft tumors analyzed by immunohistochemistry. *, *P *<* *0.05

### 3.6 Angiogenesis is enhanced by high expression levels of GNA13 in CRC tissues

α‐SMA and CD31 staining results demonstrated that there were pericytes and vascular endothelial cells in the blood vessels. There were more α‐SMA and CD31‐positive cells in GNA13 tumors in comparison with control tumors (Figure 6A), suggesting that high expression levels of GNA13 facilitate tumor angiogenesis. We next investigated the levels of proteins that are involved in tumor metastasis and angiogenesis in the sera of control and GNA13 tumor‐bearing mice. Notably, the protein levels of LOX, MMP9, and VEGF in the sera from GNA13 tumor‐bearing mice were increased compared to those in the sera from control mice (Figure 6B). Additionally, LOX, VEGF, and MMP9 levels in GNA13 tumors were markedly increased compared to those in control tumors (Figure 6C). These data demonstrate that the increased levels of those proteins in the serum were probably caused by their enhanced expression in the GNA13 tumors. These results strongly suggest that metastasis and angiogenesis are stimulated by high GNA13 expression levels in CRC via increased expression levels of MMP9, LOX, and VEGF.

**Figure 6:** GNA13 overexpression promotes angiogenesis (A) Immunofluorescent staining of CD31 (red) and α‐SMA (red) merged with nuclei (blue) in vector and GNA13 HCT116 tumors. B, VEGF, MMP9, MMP2, and LOX in sera from GNA13 tumor‐bearing mice and vector mice were analyzed by Western blotting. C, The expression of MMP9, VEGF, and LOX in GNA13 and vector tumors as assessed by immunohistochemistry

## 4 DISCUSSION

Conventional chemotherapy for CRC treatment involves combinations of cytotoxic drugs, such as 5‐fluorouracil (5‐FU), oxaliplatin, and irinotecan, and has limited efficacy and substantial side effects due to lack of specificity.^18^ Although the incidence of CRC has decreased in America, there are ethnic disparities in mortality and morbidity.^19^ It is of great necessity to develop and improve targeted therapies for the treatment of CRC.

GNA13 has recently been shown to be highly expressed in a variety of human malignancies, including gastric carcinoma, liver carcinoma, and lymphoma, and is positively correlated with tumor progression.^15^, ^20^, ^21^, ^22^ However, the role of GNA13 in CRC is unknown. Our study showed that the upregulation of GNA13 in CRC tissues was related to an exacerbated tumor grade and shorter survival. Our results also indicated that the overexpression of GNA13 in CRC promoted the proliferation of tumor cells and angiogenesis, contributing to subcutaneous tumor growth in mice.

Epithelial‐mesenchymal transition is regarded as a critical step in tumor metastasis and invasion.^23^ It is known that CRC with EMT characteristics shows more vascular invasion and metastases and has a poorer prognosis.^24^ In our study, we revealed that GNA13 expression regulates EMT in CRC cells, suggesting that GNA13 drives tumor proliferation.

We also found that overexpressing GNA13 in CRC upregulated the expression of CXCL1, CXCL2, and CXCL4, as well as chemokines with mitogenic and pro‐angiogenic activities. Therefore, GNA13 may be a key oncogenic protein in CRC. Moreover, it is crucial for angiogenesis and tumor growth because it increases the expression levels of the chemokines CXCL1, CXCL2, and CXCL4. This finding provides new information about the function of GNA13 in CRC. Our results also provided clues for developing new therapeutic drugs for CRC. Although we cannot exclude the roles of other growth factors or proteinases from our experimental conditions, it is possible that GNA13‐mediated tumor malignancy occurs mainly through activating the NF‐κB pathway. Therefore, it is necessary to understand in detail the function and the regulatory mechanisms involved in NF‐κB signaling in CRC in order to refine the effects of target therapies.

Colorectal cancer patients with increased levels of chemokines and their related receptors in ascites, plasma, and tumor tissues often have poor survival and prognosis. In addition to acting as pro‐angiogenic factors, chemokines could also act as autocrine growth factors to affect the proliferation of tumor cells.^25^ The present study revealed that the suppression of CXCL1, CXCL2, or CXCL4 in CRC cells by GNA13 overexpression significantly inhibited clonogenic growth and cell proliferation. These findings were consistent with the previous findings that CXCL4 might be a mitogenic factor that promotes cancer cell proliferation. The importance of the NF‐κB signaling pathway in CRC has been proven by its frequent activation and association with rapid cancer progression once the expression of its transcriptional targets is upregulated.^26^ A previous study also suggested an essential role of NF‐κB signaling in the regulation of chemokines, such as CXCL1 and CXCL4.^27^ Our results demonstrated that the inhibition of IKKβ and the NF‐κB p65 subunit at either the gene or protein level significantly downregulated CXCL1, CXCL2, and CXCL4 expression in CRC cells. Tumor growth, metastasis, and migration are dependent upon blood supply to the relevant tissues.^28^ Active tumor angiogenesis is linked with a short overall survival and poor prognosis in CRC patients.^28^ In addition to well‐accepted angiogenic factors, such as VEGF and platelet‐derived growth factor, the identification of novel angiogenic mediators specific to CRC is necessary.^29^ The present study used CD31 immunostaining to show that GNA13 significantly increased the tube formation of HUVECs in vitro and promoted angiogenesis in xenograft tumors. It is well known that tumor angiogenesis may be facilitated by pro‐angiogenic factors, such as VEGF, that are secreted by tumor cells; these factors can promote endothelial cell survival, migration, and proliferation to form new blood vessels.^30^, ^31^ Supporting the fact that CXCL1 and CXCL4 are potent factors with pro‐angiogenic activities and are often upregulated in ovarian cancer, our study revealed that the mRNA expression of CXCL1, CXCL2, and CXCL4 was upregulated in CRC, and the protein levels of these three chemokines were increased in the cultured medium of CRC cells.^32^ Importantly, HUVEC tube formation was abolished by the CXCR2 antagonist AZD5069 in CRC, suggesting that the upregulation of chemokines by the overexpression of GNA13 directly affected vascular endothelial growth.

In summary, our study reveals that GNA13 overexpression upregulates the expression of CXCL1, CXCL2, and CXCL4, which are chemokines involved in the IKKβ/NF‐κB pathway, and these effects are crucial for the angiogenesis and progression of CRC.

## CONFLICT OF INTEREST

None declared.

## Supporting information


** **
